The article "Genetic Manipulation of Leishmania donovani to Explore the Involvement of Argininosuccinate Synthase in Oxidative Stress Management" was retracted in 2023. Reasons: duplicated images; original data or images not available; unreliable data.

# Genetic Manipulation of *Leishmania donovani* to Explore the Involvement of Argininosuccinate Synthase in Oxidative Stress Management

**DOI:** 10.1371/journal.pntd.0004308

**Published:** 2016-03-03

**Authors:** Abul Hasan Sardar, Armando Jardim, Ayan Kumar Ghosh, Abhishek Mandal, Sushmita Das, Savita Saini, Kumar Abhishek, Ruby Singh, Sudha Verma, Ajay Kumar, Pradeep Das

**Affiliations:** 1 Division of Molecular Biology, Rajendra Memorial Research Institute of Medical Sciences, Bihar, India; 2 Institute of Parasitology and Centre for Host-Parasite Interactions, Macdonald Campus, McGill University, Quebec, Canada; 3 Department of Microbiology, All India Institute of Medical Sciences, Bihar, India; 4 Department of Biotechnology, National Institute of Pharmaceutical Education and Research (NIPER), Bihar, India; U.S. Food and Drug Administration and Center for Biologics Evaluation and Research, UNITED STATES

## Abstract

Reactive oxygen and nitrogen species (ROS and RNS) produced by the phagocytic cells are the most common arsenals used to kill the intracellular pathogens. However, *Leishmania*, an intracellular pathogen, has evolved mechanisms to survive by counterbalancing the toxic oxygen metabolites produced during infection. Polyamines, the major contributor in this anti-oxidant machinery, are largely dependent on the availability of L-arginine in the intracellular milieu. Argininosuccinate synthase (ASS) plays an important role as the rate-limiting step required for converting L-citrulline to argininosuccinate to provide arginine for an assortment of metabolic processes. *Leishmania* produce an active ASS enzyme, yet it has an incomplete urea cycle as it lacks an argininosuccinate lyase (ASL). There is no evidence for endogenous synthesis of L-arginine in *Leishmania*, which suggests that these parasites salvage L-arginine from extracellular milieu and makes the biological function of ASS and the production of argininosuccinate in *Leishmania* unclear. Our previous quantitative proteomic analysis of *Leishmania* promastigotes treated with sub-lethal doses of ROS, RNS, or a combination of both, led to the identification of several differentially expressed proteins which included ASS. To assess the involvement of ASS in stress management, a mutant cell line with greatly reduced ASS activity was created by a double-targeted gene replacement strategy in *L*. *donovani* promastigote. Interestingly, LdASS is encoded by three copies of allele, but Western blot analysis showed the third allele did not appear to express ASS. The free thiol levels in the mutant *LdASS*^-/-/+^ cell line were decreased. Furthermore, the cell viability in L-arginine depleted medium was greatly attenuated on exposure to different stress environments and was adversely impacted in its ability to infect mice. These findings suggest that ASS is important for *Leishmania donovani* to counterbalance the stressed environments encountered during infection and can be targeted for chemotherapeutic purpose to treat visceral leishmaniasis.

The article "Genetic Manipulation of Leishmania donovani to Explore the Involvement of Argininosuccinate Synthase in Oxidative Stress Management" was retracted in 2023. Reasons: duplicated images; original data or images not available; unreliable data.

## Author Summary

*Leishmania sp*. is an obligate intracellular parasite encounter toxic oxidative and nitrosative species (ROS and RNS) during infection, yet a subset of parasites infect and replicate within mammalian macrophages and eventually lead to disease symptoms. Polyamine synthesis, which is essential to counter the toxic effect of ROS and RNS, is largely dependent on the availability of L-arginine in the intracellular milieu. Argininosuccinate synthase (ASS) plays an important role as the rate-limiting step required for converting L-citrulline to argininosuccinate to provide arginine. To assess the involvement of ASS in stress management, a cell line lacking two of three *LdASS*^-/-/+^alleles, with greatly reduced ASS activity, was generated by a double-targeted gene replacement strategy in *L*. *donovani* promastigote. The free thiol levels in the *LdASS*^-/-/+^ mutant cell line were decreased. Furthermore, in L-arginine depleted medium the viability of the mutant cell line was greatly attenuated on exposure to different stress environments. The *LdASS*^-/-/+^ mutant cell line was adversely impacted in its ability to infect mice. These findings suggest that ASS is important for *Leishmania donovani* to survive in stressed environments and can be exploited as anti-leishmanial drug target.

## Introduction

Leishmaniasis represents a group of diseases caused by infection with parasites of the genus *Leishmania*, a pathogen that is transmitted by the phlebotomine sandfly [1]. *Leishmania* is an obligate intracellular parasite that infects and replicates within mammalian macrophages. It has two principal life cycle stages: the flagellated mobile promastigote that is adapted to live in the gut of the sandfly vector and an intracellular amastigote form that reside in phagolysosome of host macrophage. Promastigotes introduced during the taking of blood meal by a sandfly are rapidly phagocytized through a receptor mediated process by macrophage and once in the phagolysosome these parasites transform into an amastigote which can replicate in the harsh environment of the phagolysosome. Intracellular amastigotes are the infectious stage that cause the clinical manifestations associated with leishmaniasis, a disease characterized by various symptoms ranging from self-healing cutaneous ulcer to a potentially fatal visceral form of the disease resulting in high parasite burdens in the liver and spleen [2].

The article "Genetic Manipulation of Leishmania donovani to Explore the Involvement of Argininosuccinate Synthase in Oxidative Stress Management" was retracted in 2023. Reasons: duplicated images; original data or images not available; unreliable data.

These two life-cycle stages have differential sensitivities to reactive oxygen species (ROS) and provoke different oxidative responses in macrophage. Following the interaction with *Leishmania*, macrophages are activated and become “effector cells” that can phagocytose and destroy the unwanted guest. Macrophage activation is accompanied by the production of phagolysosomal hydrolases (e.g., proteases, nucleases, phosphatases, lipases, and esterases), the initiation of an oxidative burst, and nitric oxide (•NO) production [3–5]. The initial response marshaled by macrophages in combating internalized microbes is the respiratory burst mechanism that results in the production of superoxide reactive oxygen species [6, 7]. *Leishmania* susceptibility to ROS is dependent on the parasite stage: metacyclic promastigotes are more resistant to killing when compared to procyclic promastigotes which are particularly sensitive to superoxide and hydroxyl radicals generated from H_2_O_2_ [8–10]. A second anti-leishmanial oxidant produced by macrophages is nitrous oxide (NO) [11–13]. Unlike ROS, which are generated during phagocytosis, NO production requires macrophage activation by IFN-γ and TNF-α, cytokines linked to the killing of intracellular amastigotes [14]. In human macrophage, NO required to kill intracellular *L*. *major* amastigotes is triggered by stimulation of macrophage through the low affinity Fcε receptor, CD23 and IFN-γ [15].

Despite the robust ROS and nitrosative responses initiated by activated macrophages, a subset of metacyclic promastigotes is still able to transform into amastigotes and eventually establish an infection [16–18]. The exact mechanisms that *Leishmania* use to resist the toxic effects of ROS is not known, however, several parasite surface molecules that include, lipophosphoglycan (LPG) and glycoprotein GP63 have been found to be important in protecting parasites by scavenging toxic oxygen products or inhibit macrophage responses [19, 20]. Trypanosomes and *Leishmania* also possess trypanothione (TSH), a unique redox-cycling glutathione-spermidine conjugate, which in concert with trypanothione reductase, maintains the intracellular reducing environment in the parasite which helps counter the oxidative effects of ROS [21, 22].

Quantitative proteomic analysis of *Leishmania* promastigotes treated with sub-lethal doses of ROS, reactive nitrogen species (RNS), or a combination of both of these reagents led to the identification of several differentially expressed proteins, one of which included the argininosuccinate synthase (ASS) [23]. ASS is a key urea cycle enzyme which catalyses the rate limiting step in the conversion of L-citrulline to L-arginine. It also represents a pivotal check point in regulating L-arginine metabolism [24]. In addition, ASS also has a rate-limiting role nitric oxide (NO) synthesis [25]. ASS was down regulated in the *L*. *donovani* amastigote stage when cell division is disrupted in *centrin* null mutant cell lines, which suggests that the increased expression of ASS in amastigotes is required to maintain virulence [26, 27]. An earlier investigation in *L*. *donovani* also implicated ASS in parasite pathogenesis [28]. ASS has been purified from many species and extensively studied in humans and bacteria [29]. The *ASS* gene is well conserved between eukaryotic and prokaryotic organisms [30]. In *L*. *donovani*, seems to have been acquired by lateral gene transfer from bacteria [31]. Since the related kinetoplastid parasites *Trypanosoma brucei* and *Trypanosoma cruzi* lack an *ASS* gene. *T*. *brucei* and *T*. *cruzi* are aminotelic and are devoid of a functional urea cycle due to the absence of two urea cycle enzymes one of which is argininosuccinate synthase ASS and the other is argininosuccinate lyase (ASL) [32, 56]. Interestingly, *Leishmania* produce an active ASS enzyme, yet it has an incomplete urea cycle as it lacks an argininosuccinate lyase [28].

The article "Genetic Manipulation of Leishmania donovani to Explore the Involvement of Argininosuccinate Synthase in Oxidative Stress Management" was retracted in 2023. Reasons: duplicated images; original data or images not available; unreliable data.

L-arginine is an essential amino acid for *Leishmania* as no evidence for endogenous synthesis has been reported in these parasites, which suggests that the parasite salvages this amino acid from external sources via the high-affinity arginine transporter LdAAP3 [33] and makes the biological function of ASS and the production of argininosuccate in *Leishmania* unclear.

The protozoan parasite *Leishmania* is generally considered to be diploid, although a few chromosomes have been described to be aneuploid. In *L*. *donovani*, chromosome 23 has been reported to be trisomic [34]. Changes in chromosome copy number have been reported in various *Leishmania* species following events such as genetic manipulation of essential genes [35, 36], during in vitro growth [37], after genetic exchange [38], and following drug selection in vitro [39]. Increased gene copy number due to chromosome amplification may contribute to alterations in gene expression in response to environmental conditions in the host, providing a genetic basis for disease tropism.

In the present study we explore the role of ASS in the *Leishmania* stress management during the initial stages of infection. We used targeted gene replacement strategy to replace two of the three *LdASS* alleles which was sufficient to generate mutant *L*. *donovani* promastigote cell line (*LdASS*^-/-/+^) that surprisingly was deficient in functional ASS protein expression. Here we report that parasite viability in L-arginine depleted medium is greatly reduced on exposure to oxidative stress inducing reagents. Further the parasite burdens in livers and spleens of mice infected with the *LdASS*^-/-/+^ promastigote cell line are significantly lower indicating a role for LdASS in amastigote viability.

The article "Genetic Manipulation of Leishmania donovani to Explore the Involvement of Argininosuccinate Synthase in Oxidative Stress Management" was retracted in 2023. Reasons: duplicated images; original data or images not available; unreliable data.

## Materials and Methods

### Statement of ethic

For animal experiments, procedures were reviewed and approved (project license number -INT-88-BAS/2013) by the Animal Ethical Committee at the Rajendra Memorial Research Institute of Medical Sciences, Indian Council of Medical Research. The RMRI and ICMR follow “The Guide for the Care and Use of Laboratory Animals,” 8^th^ edition by the Institute for Laboratory Animal Research.

### Parasite cultures and bacterial strains

A cloned *Leishmania donovani* AG83 (MHOM/IN/1983/AG83) cell line was used for generation of deletion mutant and over-expressing cell lines. Promastigote were grown at 25°C in 25 cm^2^ flasks (Nunc) in RPMI-1640 media (Himedia) supplemented with 10% heat inactivated FBS (Gibco). Cultures were allowed to reach stationary phase (5–6 days post inoculation), prior to inoculation into fresh medium. Top10, DH5α and BL21 (DE3) *E*. *coli* competent cells (Invitrogen) were used to maintain plasmid constructs and for recombinant protein expression, respectively.

### Sequence alignment of ASS proteins from multiple species

The amino acid sequence of argininosucinate synthase (*ASS)* from different organisms (*L*. *donovani*, *L*. *infantum*, *L*. *major*, *L*. *mexicana*, mice and human) was retrieved from NCBI database and multiple sequence alignment was performed using CLUSTAL W software (version 2.0).

### In-vitro generation of oxidative, nitrosative and peroxynitrile stress

For the in-vitro generation of oxidative stress (ROS), nitrosative stress (RNS) and peroxynitrile stress, menadione, SNAP (S-nitroso-N-acetylpenicillamine) or mixture of both reagents were used, respectively. The sub-lethal dose of all the stress inducing reagents were previously determined [23] and doses of 5 μM menadione for oxidative stress, 300 μM SNAP for nitrosative stress and mixture of 2.5 μM menadione and 250 μM SNAP for peroxynitrile stress were used in this study. The sub-lethal doses of different stress inducing agents were determined by studying the changes in percent cell viability using MTT assay according to the manufacturer’s protocol (In-Vitro Toxicology Assay kit, MTT Based, Sigma, USA).

### Relative transcription studies of *LdASS* by semi-quantitative and quantitative real-time PCR analysis

Reverse transcription was performed using 200 μg of total RNA isolated from untreated *L*. *donovani* promastigotes or parasites treated with a mixture of menadione (2.5 μM) and SNAP (250 μM) for 15 h. cDNA was generated using an anchored oligo-dT (GenHunter; H-dT11M) protocol was used as a template for PCR amplification of the argininosuccinate synthase (*LdASS*) gene using the F1/R1 primer pair and the control transcript for α-*tubulin* using the F2/R2 primer pair (S1 Table). Products were amplified using a PCR program consisting of an initial denaturation step at 94°C for 5 min and 25 amplification cycles (94°C for 30 s, 55°C or 50°C for 30 s, and 72°C for 1 min) followed by a final extension step at 72°C for 5 min. PCR products were analyzed on a 1% agarose gel and stained with ethidium bromide. All the RT-PCR products were normalized to the α-*tubulin* RT-PCR product. These semi-quantitative data were validated by quantitative RT-PCR experiments performed in a Light CyclerR 480 (Roche) using SYBR Green (Roche) chemistry. Cycling conditions were 1 cycle at 95°C for 3 min; 40 cycles of 95°C for 15 s (denaturation), 58°C for 30 s (annealing), and 72°C for 30 s (extension). The fluorescence signal was captured at the end of each cycle using the SYBR channel (490 nm excitation and 525 nm emission wavelengths). Results are expressed as the target/reference ratio of each sample normalized by the target/reference ratio of the calibrator. Here, target/reference value of cDNA from untreated promastigotes was used as calibrator and α-*tubulin* was used as reference. The results were reported as the mean of triplicate experiments.

The article "Genetic Manipulation of Leishmania donovani to Explore the Involvement of Argininosuccinate Synthase in Oxidative Stress Management" was retracted in 2023. Reasons: duplicated images; original data or images not available; unreliable data.

### Cloning, expression, purification and generation of polyclonal anti-sera to LdASS

The coding region of full length *LdASS* gene was amplified from *L*. *donovani* genomic DNA (25 ng/μl) using F3/R3 primer pair (S1 Table). The PCR product was cloned into the *Bam*HI and *Hind*III restriction endonuclease sites of pET-28a expression vector (Novagen). Recombinant LdASS protein containing a C-terminal and N-terminal hexahistidine tag was expressed in *E*. *coli* BL-21 (DE3) cells transformed with pET-28a-*LdASS* construct. *E*. *coli* were grown to 0.6 OD^600^ and recombinant protein expression was induced with 0.75 mM IPTG for 4 h and LdASS was purified using Ni^2+^-NTA resin and the purified protein was eluted using 20 mM Tris-HCl, 1 M NaCl and 250 mM imidazole. The protein concentration was determined using Bradford reagent (Bio-Rad) and bovine serum albumin as the standard protein. Polyclonal antibody production against recombinant LdASS was performed in rabbits at the Rajendra Memorial Research Institute of Medical Sciences’ Animal Facility using two doses of 200 μg purified recombinant protein in 0.2 ml PBS emulsified with an equal volume of Freund’s complete adjuvant (Sigma, USA). Serum was isolated and titers were determined by Western blot.

The article "Genetic Manipulation of Leishmania donovani to Explore the Involvement of Argininosuccinate Synthase in Oxidative Stress Management" was retracted in 2023. Reasons: duplicated images; original data or images not available; unreliable data.

### Generation of LdASS over-expressing and down regulated *L*. *donovani* promastigote cell lines

An *LdASS* over-expressing cell line (OE) was prepared by cloning the full length *LdASS* coding region with N-terminal His-tag into the *Leishmania* specific pKSNeo vector using the *SpeI* restriction endonuclease site as described previously [28, 40] using F4/R4, F5/R5 and F6/R6 primer pairs (S1 Table). *L*. *donovani* promastigotes were transfected with this episomal expression vector (pKSNeo-*LdASS*) and the culture was maintained in RPMI-1640 medium containing 100 μg/ml G418 [41]. Similarly the N-terminal His-tag of LdASS in WT was generated as described previously [28] using F5/R5 primer pairs (S1 Table) to clone into pEXP5NT and later it was cloned in pKSNeo and then transfected into *Leishmania*.

For the generation of *Leishmania* cell line with down-regulated levels of LdASS the 5’-flanking region (902 bp) of the *LdASS* open reading frame (ORF) was PCR amplified using F7/R7 primer pair (S1 Table) containing a *Sal*I or *Hind*III restriction endonuclease site, respectively. Similarly 3’-flanking region (775 bp) was PCR amplified using F8/R8 primer pair (S1 Table) containing a *Sma*I or *Bgl*II restriction endonuclease site. Both the 5’-flanking and 3’-flanking PCR products were cloned upstream and downstream of the hygromycin (HYG) or neomycin (NEO) drug cassette respectively, in pX-63-HYG and pX-63-NEO vectors. Insertion of the 5’-flanking and 3’-flanking regions was confirmed by restriction digestion and DNA sequence analysis. Plasmids were linearized with the restriction endonuclease *Hind*III and *Bgl*II and the products (~2.72 kb for hygromycin cassette and 2.48 kb for neomycin cassette) containing both the flanking regions of *LdASS* and *HYG* or *NEO* drug selection marker were purified by agarose gel electrophoresis. Wild-type (WT, *LdASS*^+/+/+^) *L*. *donovani* promastigotes were transfected via electroporation with 5 μg of the linearized fragment (5’-*LdASS*-HYG-3’-*LdASS*) using a GenePulser XCell (Bio-Rad) system as previously described [42]. Transfected parasites were selected and maintained in RPMI-1640 culture medium containing 100 μg/ml hygromycin and heterozygous promastigotes (*LdASS*^+/+/Hyg^) cell lines were confirmed by PCR analysis. The *LdASS*^+/+/Hyg^ cell line was subjected to a second round of transfection using 5 μg of the linearized fragment 5’-*LdASS*-NEO-3’-*LdASS*. Transfected parasites were selected and maintained in RPMI-1640 liquid culture medium containing hygromycin (50 μg/ml) and G418 (50 μg/ml) and PCR analysis was employed to confirm the deletion of second wild-type *LdASS* allele. Two independent mutant *L*. *donovani* promastigote cell lines denoted as *LdASS*^-/+/+^ (where one allele was deleted) and *LdASS*^-/-/+^ (where two alleles were deleted), were chosen for further analysis. The vector control (VC) promastigote cell line was generated by transfecting wild type *L*. *donovani* promastigotes with the empty vector (pX63-HYG or pX63-NEO) without flanking region of *LdASS*.

The article "Genetic Manipulation of Leishmania donovani to Explore the Involvement of Argininosuccinate Synthase in Oxidative Stress Management" was retracted in 2023. Reasons: duplicated images; original data or images not available; unreliable data.

### Western blot analysis

The *Leishmania* promastigotes (1x10^6^ cells/ml) treated with a sub-lethal dose of 5 μM menadione, 300 μM SNAP or a combination of 2.5 μM menadione and 250 μM SNAP for 15 h were washed twice with PBS, resuspended in SDS-PAGE sample buffer and proteins were separated on a 12% SDS-polyacrylamide gel and transferred to nitrocellulose membrane. Membranes were blocked with 5% BSA and probed with rabbit anti-LdASS polyclonal antibody (1:1,000 dilution). Alkaline phosphatase conjugated secondary antibody was applied at 1:5,000 dilution and blots were developed with BCIP/NBT reagent. As a control for protein loading actin was used and blots were probed with an anti-LdACT antibody (anti-LdACT, antibody against recombinant actin proteins of *Leishmania donovani*, 1:5,000 dilution).

In another experiment, cell lysate from the wild type (WT) leishmania promastigotes (1x10^6^ cells/ml) was prepared and equal amount of lysate was loaded into the well in 12% SDS-PAGE and transferred to nitrocellulose membrane. Membranes were blocked with 5% BSA and probed with increasing concentration of rabbit anti-LdASS polyclonal antibody. Alkaline phosphatase conjugated secondary antibody was applied at 1:5,000 dilution and blots were developed with BCIP/NBT reagent.

### Biochemical characterization of *LdASS* mutant cell lines

Wildtype *L*. *donovani* promastigotes (1x 10^8^) exposed to different stress conditions were harvested and washed once in ice-cold 0.9% NaCl, then twice in ice-cold PBS and finally suspended in 125 μl lysis buffer (150 mM NaCl, 1 mM EDTA, 10 mM Tris–HCl, pH 7.5, 1% Nonidet P-40 with protease inhibitor cocktail) for 1 h on ice. Lysates were clarified (12,000 x g, 4°C, 20 min) and the protein concentration in the supernatant determined using the Bradford assay and BSA as standard (Protein Assay Kit, Bio-Rad, Hercules, CA). Lysates prepared from WT cells untreated and treated with different stress inducing reagents, were incubated with Sepharose G for 10 min to clear lysates of non-specific binding proteins and then incubated with 50% slurry (25 μl) of Ni^2+^-NTA agarose beads (Qiagen) overnight at 4°C. The Ni^2+^-NTA beads were washed three times with 500 μl lysis buffer containing 300 mM NaCl. Bound proteins were used to measure ASS activity with a modified version of the assay described by Guerreiro *et*. *al*. [43]. Briefly, proteins bound to bead (12.5 μl per reaction) were resuspended in reaction buffer (20 mM Tris-HCl, pH 7.8, 4 mM ATP, 4 mM citrulline, 4 mM aspartate, 6 mM MgCl_2_, 20 mM KCl, and 0.2 units of pyrophosphatase) in a final volume of 20 μl. Control reaction buffers lacking citrulline and aspartate were used for non-specific hydrolysis. Reactions were incubated at 37°C, and then stopped after 30 min by the addition of 300 μl volume of malachite green reagent [44]. Accumulation of inorganic phosphate was determined spectrophotometrically at 650 nm, and concentrations were interpolated from a standard curve of inorganic phosphate (Pi). Due to spontaneous release of Pi in the absence of substrates, the concentration of Pi released from these affinity purified proteins or mouse liver extracts (MLE: positive control for the reaction) were determined by subtracting the mean of the values measured in the absence of substrate from the mean values found in presence of substrate. The specific ASS activity was defined as nmoles of Pi released/μg of protein/hour. Each measurement was performed in triplicate and the mean calculated. α-methyl-DL-aspartic acid (MDLA, 5 μM) was used as inhibitor of mouse and *Leishmania* ASS enzymes [45].

The article "Genetic Manipulation of Leishmania donovani to Explore the Involvement of Argininosuccinate Synthase in Oxidative Stress Management" was retracted in 2023. Reasons: duplicated images; original data or images not available; unreliable data.

To estimate the production of argininosuccinate, reactions were run in parallel in the absence of pyrophosphatase as described by Portoles and Rubio [46]. Briefly, after 1 h incubation at 37°C, the supernatant was separated from the Ni^2+^-NTA bead pellet and subjected to reverse phase high performance liquid chromatography (HPLC). Argininosuccinate levels were analyzed by HPLC after pre-column derivatization with O-phthaldialdehyde (OPA) to convert the reaction products to fluorescent derivatives, as described by Portoles and Rubio [46]. Each measurement was performed in triplicate.

The levels of intracellular reduced thiols were measured using deproteinized *L*. *donovani* cell extracts (1x 10^8^ cells for every cell lines). The thiol content in the supernatant was measured with DTNB (Ellman’s reagent) [47] in 0.2 M Na_3_PO_4_ buffer (pH 8.0). The concentration of DTNB thiol derivatives were estimated spectrophotometrically at 412 nm. Difluoromethylornithine (DFMO, 5 μM) was used as an inhibitor of ornithine decarboxylase (ODC) and methylthiopropylamine (MTPA, 100 nM) was used as an inhibitor of spermidine synthase (SPS) [48, 49]. Each measurement was performed in triplicate.

The article "Genetic Manipulation of Leishmania donovani to Explore the Involvement of Argininosuccinate Synthase in Oxidative Stress Management" was retracted in 2023. Reasons: duplicated images; original data or images not available; unreliable data.

Polyamines (putrescine and spermidine) were identified and quantified by high performance liquid chromatography (HPLC) using a prederivatization method described by [50, 51]. Briefly, different *L*. *donovani* cell lines i.e. WT, VC, OE and *LdASS*^-/-/+^ parasites were harvested, washed twice with PBS (pH 7.4) and the cell pellet was resuspended in 5% (w/v) trichloroacetic acid overnight. The extracts were centrifuged (10,000 x*g*, 15 min) and 200 μl of supernatant was neutralized with 200 μl of a saturated NaHCO_3_ solution. The mixture was dansylated at 50°C overnight with 400 μl of a solution containing 20 mg dansyl chloride/ml in acetone (HPLC grade). The polyamines were extracted twice with toluene (Merck, HPLC grade), evaporated under nitrogen stream and the residue dissolved in 1 ml of acetonitrile (Merck, HPLC grade), prior to analysis by HPLC on a C18 reverse-phase column (Shimadzu, Japan). Dansyl polyamines were detected with a fluorescence spectrophotometer (excitation wavelength 330 nm, emission wavelength 510 nm). The peak areas, retention times were recorded and calculated by a PC Integration Pack Programme. Polyamines were expressed as nmol per 10^7^ promastigotes. There were two replicates in each test, and the data were the mean±SDs of three observations.

### Measurement of ROS level

Intracellular oxidant levels were determined using 2', 7'-dichlorodihydrofluorescein diacetate (H_2_DCFDA) (Sigma), which when oxidized becomes the highly fluorescent compound dichlorofluorescein (DCF). Levels of ROS in the different *L*. *donovani* cell lines (WT, VC, OE and *LdASS*^*-/-/+*^) treated with menadione, were monitored at various time intervals by incubating aliquots of parasite culture with 0.4 mM H_2_DCFDA for 15 min in the dark. The cells were washed with PBS (pH 7.2) and lysed with lysis buffer (1% SDS & 1% Triton X-100 in 10 mM Tris) and the fluorescence intensity of the supernatant measured using an LS55 Perkin Elmer spectrofluorimeter with an excitation wavelength of 504 nm and an emission wavelength of 529 nm and the data was expressed as relative fluorescence unit (RFU). The reagent blank was prepared with 0.4 mM H_2_DCFDA in lysis buffer. Each measurement was performed in triplicate and data expressed as mean. The fluorescence in the *L*. *donovani* cell lines were also examined by fluorescence microscopy after staining with 0.4 mm H_2_DCFDA.

### MTT assay

*Leishmania* promastigotes (1x 10^6^ cells/ml) were cultured in 24 well plates and treated with 7.5 μM menadione, 350 μM SNAP or a combination of 5 μM menadione and 300 μM SNAP and at 12 h intervals cells were harvested and viability assessed using the MTT assay (In-Vitro Toxicology Assay kit, MTT Based, Sigma, USA). Briefly, 200 μl of cell suspension containing 2 x10^5^ parasites was mixed with 20 μl of MTT solution and incubated at 25°C for 3 h. Formazen crystals were solubilized by the addition of 200 μl of MTT solubilization buffer and the optical density of the solution measured at 570 nm. To assess the importance of L-arginine in combating oxidative stress three media compositions were used, L-arginine free RPMI-1640, L-arginine free RPMI-1640 supplemented with either 50 mg/L or 200 mg/L L-arginine (Himedia). Cell viability was determined by comparing untreated to treated *L*. *donovani* cultures. Each measurement was performed in triplicate and data expressed as the mean value.

The article "Genetic Manipulation of Leishmania donovani to Explore the Involvement of Argininosuccinate Synthase in Oxidative Stress Management" was retracted in 2023. Reasons: duplicated images; original data or images not available; unreliable data.

### Murine infectivity studies

Female BALB/c (6–8 week old) were inoculated via intracardial (IC) injection with 1 X 10^7^ metacyclic stage WT, VC, OE and *LdASS*^-/-/+^ *L*. *donovani* promastigote cell lines. Four weeks post infection, mice were sacrificed and the parasite burden in spleen was quantified and expressed as Leishman-Donovan units (LDU) using the formula: LDU = [(number of parasites/1000 host nuclei) x organ (spleen) weight in milligrams (mg) [26].

### Cell viability of *L*. *donovani* amastigotes and cytokine production

Female BALB/c (6–8 week old) mice were inoculated with 4% starch solution into the intraperitoneal cavity. After 48 hr, peritoneal exudate cells (PECs) were isolated, cultured in RPMI-1640 media and grown in 6 well plate (Nunc) overnight at 37°C in CO_2_ (5%) incubator to promote adherence of macrophages. Unbound cells were removed by washing and macrophages were infected with the various *L*. *donovani* cell lines (i.e. WT, VC, OE and *LdASS*^-/-/+^) at a multiplicity of infection of 10:1 (promastigotes:macrophage) and cultures were incubated at 37°C in CO_2_ (5%)and after 24 h of infection, culture supernatant was collected and IL-10, IFN-γ, TGF-β and IL-12 cytokine levels were measured by ELISA kit (R&D system) according to the manufacturer’s protocol. Macrophage infection index for each *L*. *donovani* cell line was determined by phase contrast microscope after staining macrophage cultures with Geimsa stain.

## Results

### Primary structure analysis

Primary structure analysis of ASS proteins from phylogenetically diverse organisms revealed that it is highly conserved (>98% similarity) within *Leishmania sp*. but less conserved (~60%) when aligned with ASS sequences from the higher eukaryotes such as mice and human. ASS enzymes contain four segments (amino acids 16–27, 127–141, 278–283, and 285–290) that are highly conserved between *Leishmania*, mouse and human (Fig 1) which correspond to the nucleotide (residues 10–18, and 115–123), ATP, citrulline and an aspartate binding site. The residue at position 36 in ATP binding site is highly conserved but the nucleotide binding sites, residue 87 of citrulline binding site and residue 123 of aspartate binding site were not well conserved in the mice and human counterpart. All amino acid positions mentioned in this analysis corresponds to *Leishmania* ASS sequence.

The article "Genetic Manipulation of Leishmania donovani to Explore the Involvement of Argininosuccinate Synthase in Oxidative Stress Management" was retracted in 2023. Reasons: duplicated images; original data or images not available; unreliable data.

**Fig 1:** Sequence alignment of the *L*. *donovani*, *L*. *infantum*, *L*. *major*, *L*. *mexicana*, mouse and human argininosuccinate synthase. The predicted amino acid sequence of LdASS was aligned with other *Leishmania sp*.ASS as well as with ASS of mice and human using Clustal W software (version 2.0). The nucleotide binding domain, some conserved domain, ATP binding domain, aspartate binding domain, citrulline binding domain are shown in box.

### *L*. *donovani* argininosuccinate synthase (*LdASS*) is up-regulated in response to stress

To study the temporal effect of stress inducing agents on the expression of *LdASS* both semi-quantitative and real-time PCR analysis were performed to measure the levels of mRNA following treatment of promastigotes with a mixture of menadione and SNAP. The *LdASS* mRNA was up-regulated ~2.4 fold when analyzed in semi-quantitative RT-PCR (Fig 2A and 2B) whereas in real-time PCR, it was up-regulated 4.8 fold (Fig 2C).

**Fig 2:** Relative expression levels of the *L*. *donovani* ASS in response to oxidative stress. Wild type (WT) *L*. *donovani* parasites were treated with a mixture of 2.5 μM menadione and 250 μM SNAP and the relative *LdASS* mRNA expression levels were measured by semi-quantitative RT-PCR, (A) using promastigotes exposed to an oxidative (O) and nitrosative (N) stress or unstimulated (UNS) control cell. Amplification of a DNA fragment corresponding to *α-tubulin* was used as the loading control. B) Densitometry analysis of RT-PCR products for *LdASS* and *α-tubulin* was performed on ethidium bromide stained agarose gels. Bar diagram showing the *LdASS* mRNA level was increased by ~2.4-fold in O+N stress cells. C) Real-Time PCR analysis was performed to quantify the *LdASS* and *α-tubulin* mRNA levels following oxidative and nitrosative stress (O+N) treatment or unstimulated controls. Bar diagram showing that the ASS mRNA level was increased ~4-fold in O+N stress cells. Each measurement was performed in triplicate and data are expressed as the mean. Vertical lines on top of the bars represent S.E. (standard error) values and star symbol above the vertical lines denotes significant changes with P<0.005.

### Characterization of *L*. *donovani* mutant cell lines

To further examine the role of argininosuccinate synthase in combating the reactive oxidative stresses encountered by promastigotes during macrophage invasion, four *L*. *donovani* mutant cell lines were used. These included, wild-type (WT, *LdASS*^+/+/+^), vector control (VC) which was transfected with empty vector, an LdASS over-expresser cell line (OE) transfected with the pKSNeo-*LdASS* plasmid, a heterozygous cell line (*LdASS*^-/+/+^) in which one *LdASS* allele was deleted by targeted gene replacement with the 5’flank-*LdASS*-pX-63-HYG-3’flank-*LdASS* construct, and a second heterozygous cell line (*LdASS*^-/-/+^) in which two *LdASS* alleles were deleted 5’flank-*LdASS*-pX-63-HYG-3’flank-*LdASS* and the 5’flank-*LdASS*-pX63-NEO-3’flank-*LdASS* constructs (Fig 3A).

The article "Genetic Manipulation of Leishmania donovani to Explore the Involvement of Argininosuccinate Synthase in Oxidative Stress Management" was retracted in 2023. Reasons: duplicated images; original data or images not available; unreliable data.

**Fig 3:** Targeted gene replacement of *LdASS* alleles, expression and purification of recombinant *LdASS* protein. A) Schematic representation of the *LdASS* locus and the plasmid constructs used for gene replacement experiments is illustrated. B) PCR analysis of the -amplified products of *LdASS* gene. Lanes: PCR with genomic DNA from WT, *LdASS*^-/+/+^ mutant and *LdASS*^-/-/+^ mutant cell lines to amplify full length (1250 bp) *LdASS* gene (*lanes* 1–3), molecular weight marker (M), PCR with genomic DNA from WT, *LdASS*^-/+/+^ mutant and *LdASS*^-/-/+^ mutant using F7/R8 primer pairs (S1 Table). External forward (F7) and reverse (R8) primers were designed from 902 bp upstream of the *LdASS* gene and 775 bp downstream of the stop codon of the gene, respectively. The expected size of *LdASS*, HYG and NEO gene PCR products were 2.93, 2.72 and 2.48 kb, respectively (lanes 5–7). C) PCR amplified products using primers (F9/R9, F10/R10, F11/R11 and F12/R12) (S1 Table) designed from the upstream and downstream sequences of 5’-flanking region and 3’flanking region respectively (outside of the gene deletion construct) and internal region of the two genes used as selectable marker i.e. hygromycin phosphotransferase (*HPT* for HYG resistance) present in pX-63-HYG and neomycin phosphotransferase (*NPT* for neomycin resistance) present in pX-63-NEO plasmid vectors respectively. The PCR image showed the presence of two bands correspond to 1100 bp and 913 bp (5’flank-*LdASS*-pX-63-HYG-3’flank-*LdASS* construct) in *LdASS*^-/+/+^ cell line (lane 1) and four bands correspond to 1100 bp and 913 bp (5’flank-*LdASS*-pX-63-HYG-3’flank-*LdASS* construct); 1030 bp and 833 bp (5’flank-*LdASS*-pX-63-NEO-3’flank-*LdASS* construct) in *LdASS*^-/-/+^ cell line (lane 2). In WT cell line no bands were detected (lane 3). Lane M containing the molecular weight marker loaded. D) SDS-PAGE analysis for the expression of recombinant LdASS protein. Lane 1, molecular weight marker; lane 2, -IPTG; lane 3, + IPTG (IPTG induction for 4 hours). E) SDS-PAGE analysis of purified recombinant LdASS protein. Lanes 1–3, purified protein; lane 4, molecular weight marker. F) Western blot shows the relative expression levels of LdASS and actin in the various wild type and mutant *L*. *donovani* promastigote cell lines. G) Bar diagram showing expression level of LdASS protein in different cell lines. Each measurement was performed in triplicate and data are expressed as the mean. Vertical lines on top of the bars represent s.e. values and star symbol above the vertical lines denotes significant changes with P<0.005.

The article "Genetic Manipulation of Leishmania donovani to Explore the Involvement of Argininosuccinate Synthase in Oxidative Stress Management" was retracted in 2023. Reasons: duplicated images; original data or images not available; unreliable data.

The genotype of the various *L*. *donovani* promastigote cell lines was confirmed by PCR analysis using primer pairs to amplify, the *LdASS* ORF, and the disrupted locus using external primers that were complementary to a region 902 bp up-stream and 775 bp down-stream of *LdASS* ORF, respectively. A single ~1.25 kb band corresponding to the *LdASS* ORF was observed for the WT, *LdASS*^-/+/+^, and *LdASS*^-/-/+^ (Fig 3B). The band intensity for the wild-type cell line was ~two-fold higher than *LdASS*^-/+/+^ and ~four-fold higher than the *LdASS*^-/-/+^ cell line. Surprisingly, for *LdASS*^-/-/+^ it was anticipated that *LdASS* was encoded by two alleles that after two rounds of targeted gene replacement would eliminate the gene, however a ~1.25 kb was still detected in this cell line (Fig 3B). To further validate the rearrangement of the *LdASS/ldass* loci, PCR experiments were performed using primers to the 5’-flanking and 3’-flanking regions. The size of the expected PCR products for these experiments was a ~2.93 kb for the wild type *LdASS* locus, a ~2.72 and ~2.48 kb fragments for loci containing a *HYG* and *NEO* drug cassette, respectively (Fig 3B). An ~2.93 kb product was observed for the wild type, *LdASS*^-/+/+^ and *LdASS*^-/-/+^ cell lines (Fig 3B). The presence of a ~2.93 kb fragment in the *LdASS*^-/-/+^ cell line, although significantly diminished in intensity when compared to the wild type cell line, suggested that the *LdASS*^-/-/+^ mutant cell line retained a copy of *LdASS* despite two rounds of targeted gene replacement. DNA from the *LdASS*^-/+/+^ cells gave rise to two bands with sizes of ~2.93 kb and ~2.72 kb, but for *LdASS*^-/-/+^ cell line three bands corresponding to the sizes ~2.93 kb, ~2.72 kb and ~2.48 kb were observed. In the case of *LdASS*^-/+/+^ cell line, as expected after PCR with external primers, two bands; one containing *LdASS* gene (~2.93 kb) and other containing the HYG gene (~2.72 kb) were observed. In the case of *LdASS*^-/-/+^ cells an extra single band corresponding to ~2.48 kb was expected as the second *LdASS* allele was expected to be replaced by *NEO* gene. But surprisingly two bands; one corresponding to ~2.93 kb and one corresponding to ~2.48 kb were observed. An interesting fact was that the intensity of the ~2.93 kb band in the *LdASS*^-/-/+^cell line was lower than the band observed in *LdASS*^-/+/+^ cell line (Fig 3B). A result consisted with the chromosome carrying the LdASS gene being triploid.

The article "Genetic Manipulation of Leishmania donovani to Explore the Involvement of Argininosuccinate Synthase in Oxidative Stress Management" was retracted in 2023. Reasons: duplicated images; original data or images not available; unreliable data.

Another PCR analysis performed with primers (F9/R9, F10/R10, F11/R11 and F12/R12) (S1 Table) designed from the upstream and downstream sequences of 5’Flanking and 3’flanking region respectively (outside of the gene deletion construct) and internal region of the two genes used as selectable marker i.e. hygromycin phosphotransferase (*HYG* resistance) present in pX-63-*HYG* and neomycin phosphotransferase (*NEO* resistance) present in pX-63-*NEO* plasmid vectors respectively. The PCR analysis showed the presence of two bands correspond to ~1100 bp and ~913 bp (5’flank-*LdASS*-*HYG*-3’flank-*LdASS* construct) in *LdASS*^-/+/+^ cell line and four bands correspond to ~1100 bp and ~913 bp (5’flank-*LdASS*-*HYG*-3’flank-*LdASS* construct); ~1030 bp and ~833 bp (5’flank-*LdASS*-*NEO*-3’flank-*LdASS* construct) in *LdASS*^-/-/+^ cell line. Again this result confirmed that in *LdASS*^-/+/+^ cell line, one *LdASS* allele was deleted but in *LdASS*^-/-/+^ cell line, two *LdASS* alleles were deleted. In WT cell line no bands were detected (Fig 3C).

### Characterization of the *L*. *donovani* LdASS over-expresser

To further validate the phenotype of the various *LdASS/ldass L*. *donovani* cell lines, Western blot analysis was performed using LdASS specific polyclonal antisera to examine the levels of this enzyme. First the expression of LdASS in *L*. *donovani* cell lysate was determined in Western blot (S1 Fig). Interestingly, another Western blot analysis showed that over-expressed band and a faint band (down-regulated expression) corresponding to LdASS protein was detected in case of OE cell line and *LdASS*^-/+/+^ cell line respectively. Surprisingly, no band was detected in case of *LdASS*^-/-/+^ cell line (Fig 3F and 3G). This Western blot analysis suggested that the *LdASS*^-/-/+^ cell line despite having an *LdASS* copy fails to express detectable levels of LdASS.

To estimate the levels of LdASS in various *LdASS/ldass* cell lines enzymatic assays were performed. Exposing the WT cell line to the stress inducing reagents, menadione (oxidative stress) or a mixture of menadione and SNAP induced a ~1.8-and ~1.5-fold increase in enzymatic activity, respectively (Fig 4A). Treatment of the lysate from WT cell line with 5 mM α-methyl-DL-aspartic acid, a specific inhibitor of ASS resulted in ~100% decrease in LdASS (Fig 4A).

The article "Genetic Manipulation of Leishmania donovani to Explore the Involvement of Argininosuccinate Synthase in Oxidative Stress Management" was retracted in 2023. Reasons: duplicated images; original data or images not available; unreliable data.

**Fig 4:** Assay of enzyme activity, argininosuccninate production, western blot analysis, assay of reduced thiol pool and polyamine level. A) ASS enzyme activity of WT *L*. *donovani* cell line under stress conditions. Exposing the WT cell line to the stress inducing reagents, menadione (oxidative stress) or a mixture of menadione and SNAP induced a ~1.8-and ~1.5-fold increase in enzymatic activity, respectively was observed. About 100% enzymatic activities were blocked when WT cells were incubated with 5 mM α-methyl-DL-aspartic acid (MDLA), (a specific inhibitor of ASS). B) Bar-graph showing the amount of ASA produced in different in WT *L*. *donovani* exposed to different stress inducing reagents. The argininosuccinate levels were increased ~1.5-fold after exposure to different stress inducing reagents in comparison to WT cell line, whereas the level of argininosuccinate was decreased to the level of blank in presence of inhibitor (5 mM MDLA). C) Western Blot image of LdASS of wild type and OE cell lines. Left panel-under different stress conditions i.e. menadione (M), SNAP (S), combination of SNAP and menadione (S+M). Right panel (lanes 5–6) L-arginine limiting conditions after *L*. *donovani* cells were cultured in L-arginine free medium for two successive generations. D) Densitometry analysis of the Western Blot results. E) Bar-graph showing the amount of reduced thiol pool in WT, OE and *LdASS*^-/-/+^ cell lines under different stress conditions and in presence of two different inhibitors of enzymes involved in polyamine biosynthesis pathway. The reduced thiol level was found to be decreased in *LdASS*^-/-/+^ cells by ~3-fold compared to WT and OE cell lines, which were further decreased when exposed to different type of stress. DFMO and MTPA were used as inhibitor of ornthine decarboxylase (ODC) and spermidine synthase (SPS) respectively. Reduced thiol level was found to be decreased in *LdASS*^-/-/+^ cell line and under stress conditions. F) Bar-graph showing the relative level of two polyamines i.e. putrescine and spermidine in different *L*. *donovani* cell lines (WT, VC, OE and *LdASS*^-/-/+^). The level of both the polyamines in the *LdASS*^-/-/+^ was found to be decreased by ~4 fold compared to WT parasites whereas ~2.4 fold increased level was observed in OE parasites compared to WT parasites. Each measurement was carried out in triplicate and data are expressed as the mean. Vertical lines on top of the bars represent s.e. values and star symbol above the vertical lines denotes significant changes with P<0.005.

The article "Genetic Manipulation of Leishmania donovani to Explore the Involvement of Argininosuccinate Synthase in Oxidative Stress Management" was retracted in 2023. Reasons: duplicated images; original data or images not available; unreliable data.

### LdASS expression under oxidative stress and limiting-arginine environments

Western blot analysis showed that in response to oxidative stimuli both WT and LdASS OE cell lines up-regulated the expression of LdASS. The WT cell line treatment with SNAP, showed only a minor ~1.4-fold increase in LdASS; while menadione or a mixture of SNAP/menadione triggered a ~4.2-fold and ~3.8-fold increase in LdASS, respectively (Fig 4C and 4D). A similar response was also observed with the LdASS OE cell line which showed a ~1.6-fold, ~3.6-fold, and ~3-fold up-regulation following treatment with SNAP, menadione, or a combination of both stress inducing compounds, respectively (Fig 4C and 4D). In L-arginine free RPMI-1640 supplemented with 50 mg/L L-arginine, the expression of LdASS protein was up-regulated by~3-fold and ~4-fold for the WT and OE cell lines, respectively. Interestingly, when RPMI-1640 medium was supplemented with 200 mg/L of L-arginine the expression levels LdASS decreased by ~1.6- and ~2.5-fold for WT and OE cell lines compared to 50 mg/L L-arginine supplementation, respectively (Fig 4C and 4D).

### Argininosuccinate production, polyamine level and intracellular thiol content are decreased in LdASS down regulated mutant cell line

The final product of the enzymatic reaction catalyzed by LdASS, argininosuccinate, was measured using high pressure liquid chromatography assay. The argininosuccinate levels were increased ~1.5-fold after exposure to different stress inducing reagents in comparison to WT cell line (Fig 4B); whereas the level of argininosuccinate was decreased to background levels in the presence of the inhibitor MDLA (5 mM) (Fig 4B).

Reduced thiol levels were measured in the different *L*. *donovani* mutant cell lines using a spectrophotometric assay. Thiol levels in *LdASS*^-/-/+^ cells were ~3-fold lower when compared to WT and OE cell lines. Exposure of *Leishmania* promastigotes to oxidative stress inducing agents (menadione, SNAP and mixtures of menadione and SNAP) decreased the thiol levels in all lines when compared to the unstimulated cells (Fig 4E). Difluoromethylornithine (DFMO), was used an inhibitor of ornithine decarboxylase (ODC) and methylthiopropylamine (MTPA) was an inhibitor of spermidine synthase (SPS). Decreased thiol levels were observed in the DFMO or MTPA treated cells compared to unstimulated cells within each individual cell lines i.e WT, OE and *LdASS*^-/-/+^ (Fig 4E).

Polyamines are the major source of precursors for the synthesis of trypanothione, which is ultimately involved in regulating the stress response in *L*. *donovani* parasites [52, 53]. The level of two important polyamines i.e. putrescine and spermidine in different *L*. *donovani* cell lines i.e. WT, VC, OE and *LdASS*^-/-/+^ were measured by HPLC. The level of both polyamines in the *LdASS*^-/-/+^ was found to be decreased by ~4 fold compared to WT parasites whereas ~2.4 fold increased level was observed in OE parasites compared to WT parasites (Fig 4F).

The article "Genetic Manipulation of Leishmania donovani to Explore the Involvement of Argininosuccinate Synthase in Oxidative Stress Management" was retracted in 2023. Reasons: duplicated images; original data or images not available; unreliable data.

### ROS levels were increased in LdASS down regulated mutant cell line after exposure to menadione

ROS level in different *L*. *donovani* cell lines (WT, VC, OE and LdASS^-/-/+^) were studied both by spectrofluorometry and fluorescence microscopy. Promastigotes were treated with menadione and then incubated with H_2_DCFDA to estimate ROS level. This approach showed that ROS level were decreased by ~1.9-fold in OE cells whereas levels were increased by ~1.8-fold in LdASS down regulated cells (*LdASS*^*-/-/+*^) when compared to WT cells (Fig 5A). Fluorescence microscopy showed a greater fluorescence intensity in *LdASS*^*-/-/+*^cells whereas a lower intensity was detected in OE cells compared to WT cells (Fig 5B). These results correlated with the spectrofluorometry data.

**Fig 5:** Measurement of ROS level. ROS level in different *L*. *donovani* cell lines (WT, VC, OE and LdASS^-/-/+^) were determined both by spectroflurometry and fluorescence microscopy using H_2_DCFDA. The promastigotes were first treated with menadione and incubated with H_2_DCFDA for the estimation of ROS level. A) The ROS level was found to be decreased by ~1.9 fold in OE cells whereas increased by 1.8 fold in LdASS down regulated cells (*LdASS*^*-/-/+*^) compared to WT cells. Each measurement was performed in triplicate and data are expressed as the mean. Vertical lines on top of the bars represent s.e. values and star symbol above the vertical lines denotes significant changes with P<0.005. B) The fluorescence microscopy images showed that greater fluorescence intensity in LdASS down regulated cells whereas lower intensity in OE cells compared to WT cells.

### Parasite viability under stress environments was dependent on L-arginine availability

WT, OE and *LdASS*^-/-/+^ parasites cultured in L-arginine free RPMI-1640, L-arginine free RPMI-1640 supplemented with 50mg/L or 200 mg/L L-arginine, and dialyzed FBS then exposed to stress inducing reagents i. e. 7.5 μM menadione, 350 μM SNAP, or a mixtures of 5 μM menadione/300 μM SNAP to generate peroxynitrile stress. In L-arginine free media the cell viability for WT, OE and *LdASS*^-/-/+^ cell lines was decreased to ~51%, ~59% and ~35%, respectively in unstimulated cells (Fig 6A,6B and 6C) after 48 h in complete RPMI-1640 medium. Whereas following treatment of these cell lines with menadione, SNAP or mixture of menadione and SNAP decreased cell viability of the WT, OE and *LdASS*^-/-/+^ cell lines to ~8–10%, ~16–20% and ~0.9–3%, respectively after 48 h incubation (Fig 6A, 6B and 6C). In L-arginine restricted medium (50 mg/L), cell viabilities were increased to ~98% for unstimulated cells lines, whereas cell lines treated oxidative stress inducing compounds had viabilities of ~10–20%, ~20–40% and ~5–12% at 48 h (Fig 6D,6E and 6F). Supplementing the RPMI-1640 media with 200 mg/L of arginine resulted in on modest increase in cell viability to ~20–37%, ~25–60% and ~10–25% of the WT, OE and *LdASS*^-/-/+^ cell lines, respectively at 48 h in (Fig 6G, 6H and 6I). The increase in cell viability upon increase in L-arginine concentration in the media suggest that optimum L-arginine concentration in the media is required to maintain the parasite cell viability.

The article "Genetic Manipulation of Leishmania donovani to Explore the Involvement of Argininosuccinate Synthase in Oxidative Stress Management" was retracted in 2023. Reasons: duplicated images; original data or images not available; unreliable data.

**Fig 6:** Viability of *LdASS* mutant cell lines under nutrient restricted and replete conditions. WT, OE and *LdASS*^-/-/+^ parasites were cultured in L-arginine free RPMI-1640, L-arginine free RPMI-1640 supplemented with 50 mg/L L-arginine, L-arginine free RPMI-1640 supplemented with 200 mg/L L-arginine. Simultaneously the parasites were exposed to sub-lethal doses of stress inducing reagents i. e. menadione (M) for oxidative stress, SNAP (S) for nitrosative stress and mixtures of both menadione and SNAP for peroxynitrile stress (M+S) and the cell viability was determined using the MTT assay. Percent cell viability of WT, OE and *LdASS*^-/-/+^ cells in complete RPMI-1640 media; (A, B and C), L-arginine depleted RPMI-1640 medium, (D, E and F), in RPMI-1640 medium supplemented with 50 mg/L L-arginine (G, H and I) in L-arginine free medium supplemented with 200 mg/L.The % cell viability of unstimulated *L*. *donovani* parasite (UNS) was taken as control in each set. Each measurement was performed in triplicate and data are expressed as the mean.

### Mutant *LdASS*^-/-/+^parasites have reduced viability *in vivo* and *ex vivo*

Infection studies in BALB/c mice were performed to determine the role of LdASS expression on *Leishmania* parasite survival. BALB/c mice infected with WT, VC, OE or *LdASS*^-/-/+^ promastigotes were sacrificed after 4 weeks and the parasite loads in the spleen quantified. The parasite burdens were ~4-fold for the *LdASS*^-/-/+^ cell line but showed a ~2.3-fold increased in OE cell line when compared to the wild type and vector control parasites (Fig 7A). Phase contrast microscopy of murine peritoneal macrophages infected with different *L*. *donovani* cell lines (WT, VC, OE and *LdASS*^*-/-/+*^) showed the amastigote viability inside the macrophages (Fig 7B). These data confirm that the capacity of *L*. *donovani* parasites to metabolize arginine is critical for viability.

The article "Genetic Manipulation of Leishmania donovani to Explore the Involvement of Argininosuccinate Synthase in Oxidative Stress Management" was retracted in 2023. Reasons: duplicated images; original data or images not available; unreliable data.

**Fig 7:** Infectivity of *LdASS* mutants in the murine model. A) BALB/c mice were infected with WT, VC, OE and *LdASS*^-/-/+^ cell lines of *L*. *donovani*. After four weeks infected mice were sacrificed and parasite load was determined by counting the no. of amastigotes per100 macrophages (Mϕ) in spleen. The parasite burden in spleen was found to decrease by ~4 fold in *LdASS*^-/-/+^ cell line but increased by ~2.3-fold in OE cell line compared to WT and VC cell lines. B) Phase contrast microphotograph after Geimsa staining of PECs containing murine peritoneal macrophages infected with different *L*. *donovani* cell lines (WT, VC, OE and *LdASS*^*-/-/+*^). C & D) IL-12, IFN-γ, IL-10 and TGF-β Cytokine level were measured in murine peritoneal macrophages infected with different *L*. *donovani* cell lines (WT, VC, OE and *LdASS*^-/-/+^). In the *LdASS*^-/-/+^ parasites, the IL-12 and IFN-γ were increased whereas IL-10 and TGF-β were decreased compared to WT parasites. Each measurement was performed in triplicate and data are expressed as the mean. Vertical lines on top of the bars represent s.e. values and star symbol above the vertical lines denotes significant changes with P<0.05.

### IL-10 and TGF-β was decreased whereas IL-12 and IFN-γ were increased in PEC derived macrophages infected with *LdASS*^-/-/+^ parasites

In general during active visceral leishmaniasis the level of disease promoting cytokines are up-regulated over host protective cytokines. With the different *L*. *donovani* cell lines, i.e. WT, VC, OE or *LdASS*^-/-/+^, the levels of IL-12 and IFN-γ (host protective) and, IL-10 and TGF-β (disease promoting) were measured by ELISA. In the *LdASS*^-/-/+^ parasites, the IL-12 and IFN-γ were increased whereas IL-10 and TGF-β were decreased compared to WT parasites (Fig 7C and 7D).

## Discussion

In previous quantitative proteomic studies we showed that along with other redox homeostasis proteins, LdASS was found to be up-regulated by ~1.5–2 fold [23]. Furthermore, expression studies at the mRNA as well as protein level demonstrated an up-regulated expression of ASS in amastigote stage compared to promastigote stage [27].

Phylogenic analysis of the LdASS, revealed that this urea cycle enzyme is present prokaryotes and most higher eukaryotes. ASS is also found in *Leishmania* but not in other kinetoplastid members that also cause human disease. It is interesting to speculate that *Leishmania* may have acquired the LdASS by lateral transfer from bacteria [31, 53] or it was lost in ancestral trypanosomes after divergence of *Leishmania* as suggested for other genes i.e. *Leishmania* phenylalanine hydroxylase (PAH) [54]. Sequence alignment of ASS proteins from multiple species revealed that it is well conserved within the *Leishmania sp*. but exhibits less homology with enzyme from the higher eukaryotic organism like mice and human. Our analysis suggests that these sequence variation may be exploited for development of specific inhibitor against *L*. *donovani* ASS (Fig 1).

The article "Genetic Manipulation of Leishmania donovani to Explore the Involvement of Argininosuccinate Synthase in Oxidative Stress Management" was retracted in 2023. Reasons: duplicated images; original data or images not available; unreliable data.

The up-regulated expression of ASS at the mRNA level as observed by semi-quantitative and real time PCR experiments was correlated with our previous quantitative proteomics data [23]. Since LdASS was over-expressed upon exposure to oxidative, nitrosative or the combination of both stress agents compared to untreated wild type parasites, we speculated that LdASS has a role in stress tolerance like other stress related enzymes [21, 22, 55 and 56]. Our PCR results with external primers as well as gene specific primers (designed from the *LdASS* ORF) showed that two rounds of targeted gene replacement were not sufficient to displace all the LdASS alleles and suggested the presence of an extra *LdASS* allele in *Leishmania* genome. The possibility of an extra allele is supported by previous observations where clones retained a native chromosomal copy of the ASS gene even after generation of knock-out cell line [28] and deep sequencing results indicated that chromosome 23 (which contains the ASS gene) of *Leishmania donovani* is trisomic [34].

Western blot analysis using polyclonal sera failed to detect expression of LdASS in the *LdASS*^-/-/+^ mutant cell line. This result suggested that even though there is an extra copy of *LdASS*; it failed to produce notable levels of functional protein expression.

Further characterization of *L*. *donovani* promastigote cell lines (WT, OE and *LdASS*^-/-/+^) was carried out to examine the phenotypic effect of the gene deletion under stress environments and L-arginine limiting environments. When WT cells were exposed to different stress inducing reagents, increased argininosuccinate synthase activity was detected in all the stress environments compared to unexposed WT *L*. *donovani* cell line which suggests that the possible involvement of ASS in stress management.

The enzymatic activity of LdASS was confirmed using specific inhibitor the α-methyl-DL-aspartic acid (MDLA) [44, 57, 58] and by HPLC identification of argininosuccinic acid (ASA) in the reaction products catalyzed by WT *L*. *donovani* cells exposed to different stress inducing reagents [44]. ASS activity was increased when WT *L*. *donovani* promastigotes were exposed to different stress inducing reagents. The inability of MDLA to block LdASS during *in vivo* condition as shown in previous study [28] opens up a new window for designing and synthesizing novel specific inhibitor against LdASS.

The article "Genetic Manipulation of Leishmania donovani to Explore the Involvement of Argininosuccinate Synthase in Oxidative Stress Management" was retracted in 2023. Reasons: duplicated images; original data or images not available; unreliable data.

The final product of the enzymatic reaction catalyzed by ASS is argininosuccinic acid (ASA). The ASA level was found to be increased when WT *L*. *donovani* cells were exposed to different stress inducing reagents which co-relates with the enzymatic activity data.

*Leishmania* parasites are dependent on extracellular L-arginine availability for optimal growth. As the commercially available RPMI-1640 contains about 200 mg/L L-arginine (Himedia), we have considered L-arginine free RPMI-1640 supplemented with 200 mg/L L-arginine to match up the optimal L-arginine concentrations present in the growth media. We have used another media where L-arginine free RPMI-1640 was supplemented with 50 mg/L L-arginine to observe the effect of L-arginine availability on the expression on LdASS protein. The western Blot results showed that the LdASS was up-regulated when there is a low availability of L-arginine in the media (50mg/L) whereas this up-regulated expression of LdASS was decreased when L-arginine availability was increased to 200 mg/L in the media (Fig 4C, Lane 5 and 6, and 4D).

To counterbalance an oxidative environment that would be encountered by *Leishmania* in the macrophage phagosomal compartment it is postulated that high levels of reduced thiols would be essential for parasite viability in the mammalian host [21, 22]. Unlike other eukaryotes the primary reduced thiol found in kinetoplastids is reduced trypanothione instead of glutathione [21, 22]. Thiol level in *LdASS*^-/-/+^ cells was ~3-fold lower when compared to WT and OE cell lines. Exposure of *Leishmania* promastigotes to oxidative stress inducing agents (menadione, SNAP and mixtures of menadione and SNAP) or DFMO or MTPA a decrease in reduced thiol level was observed in case of every cell lines i.e. WT, OE and *LdASS*^-/-/+^ compared to unstimulated cells of that particular cell line. We have also observed that in *LdASS*^-/-/+^ parasites the level polyamines like putresciene and spermidine were decreased compared to WT parasites (Fig 4F). Moreover the ROS level was also found to be increased in *LdASS*^-/-/+^ parasites compared to WT parasites (Fig 5A and 5B). These results suggested that these inhibitors predominantly affected the glutathione or trypanothione level and *LdASS*^-/-/+^ parasites were susceptible to different type of stress which *Leishmania* parasite probably encounters during early stage of infection or during transformation from promastigote to amastigote. The inhibitor study suggests that the synthesis of trypanothione is necessary to maintain the reduced thiol level to counterbalance the increased ROS level which correlated with previous study [21, 22].

The article "Genetic Manipulation of Leishmania donovani to Explore the Involvement of Argininosuccinate Synthase in Oxidative Stress Management" was retracted in 2023. Reasons: duplicated images; original data or images not available; unreliable data.

Previous studies suggested that an incomplete urea cycle occurs in *Leishmania sp*. and the product of the enzymatic reaction catalyzed by ASS i. e. argininosuccinate (ASA) serves another purpose as the next gene of the urea cycle pathway is absent [59]. L-arginine is an essential amino acid for *Leishmania* growth [60]. It was also been shown that aspartate and citrulline could not substitute for arginine [28]. Our results suggested that *LdASS*^-/-/+^ (ASS down regulated parasites) were more susceptible to stress and the cell viability of *L*. *donovani* is largely dependent on L-arginine availability in the intracellular milieu (Fig 6). The intracellular L-arginine pool is maintained with the help of members of the y+ transmembrane family of proteins responsible for cationic amino acid (CAT) uptake by amino acid permease (LdAAP3), highly specific for arginine as its transport is not inhibited by other amino acids or arginine-related compounds [61, 33].

LdASS appears to be a vital component for *Leishmania* infectivity. Macrophage and murine infection studies showed that the down-regulation of LdASS dramatically decreased the survival of amastigote in peritoneal macrophage and splenic parasite burdens when compared to WT and VC parasites. In general, leishmaniasis is distinguished by mixed Th1 and Th2 response with a positive balance towards Th2 response, which is characterized by increased production of IL-10 as well as IL-4 [62]. Previous investigation shown that the proinflammatory cytokines like IL-12 and IFN-γ were upregulated upon in vitro infection of macrophages with live attenuated *L*. *donovani* parasites compared to that with wildtype [WT] parasites [26]. It is now well established that in leishmaniasis protective immunity is achieved when Th1 response, characterized by increased levels of IFN-γ and IL-12, dominates over Th2 response [63]. So, during active visceral leishmaniasis the level of disease promoting cytokines are up-regulated over host protective cytokines. Macrophages infected with LdASS-/-/+ parasites, the IL-12 and IFN-γ were increased whereas IL-10 and TGF-β were decreased compared to WT parasites. This cytokine data suggests that due to down regulation of *LdASS*, the host protective cytokines were increased over the disease promoting cytokines, which correlates with microscopy data where less amastigote viability was observed inside the infected macrophages. Impaired viability of the mutant cell lines allows the host to mount a protective response that promotes the clearance.

The article "Genetic Manipulation of Leishmania donovani to Explore the Involvement of Argininosuccinate Synthase in Oxidative Stress Management" was retracted in 2023. Reasons: duplicated images; original data or images not available; unreliable data.

*L*. *donovani* lacks the argininosuccinate lyase, so urea cycle in this parasite is incomplete. So, the fate of arginiosuccinate (AS) produced by LdASS is unclear and probably there are some undocumented events in the infected macrophage or in an infected mouse that account for the altered virulence of ASS over expressing or down-regulating *L*. *donovani* cell lines. There may be alternative way to synthesize polyamine from the AS during exposure to stress environments. L-arginine (L-arg) up take by macrophages via cationic amino acid transporter (CAT). This L-arginine pool is further taken up parasitoforus vacuole (PV) and amastigote (AM) subsequently by other different amino acid transporter (AAT). L-arginine pool can be utilized by two different pathways. In macrophages nitric oxide (NO) is produced from L-arginine when it is cleaved by NOS2 by two step mechanism. Due to action of NO parasite clearance occurs. In another side, in amastigotes L-ornithine is synthesized from L-arginine pool by arginase. Polyamine is produced from this L-ornithine via polyamine biosynthesis pathway. These polyamines can counterbalance the stress and parasite growth is favored. During exposure to stress environments or L-arginine deficiency, argininosuccinate (AS) is produced from citruline and aspartate by argininosuccinate synthase (LdASS). This AS can enters PV and subsequently Mϕ and produced L-arginine by argininosuccinate lyase (ASL) of macrophage origin. This L-arginine can further taken up the amastigote and utilized by polyamine biosynthesis pathways to produce different polyamines for counterbalancing the stress.

In this study we wanted to investigate is there any link between ASS up-regulation, stress management and amastigote cell viability? The major observations steaming from this work include a) ASS was up-regulated under different stress environments both RNA and protein level, b) The mutant *LdASS*^-/-/+^ *L*. *donovaani* cells have reduced enzymatic activity and lower level of reduced thiol, c) reduction in parasite viability as well as rate of infection in mice in case of mutant *LdASS*^-/-/+^ cells. In a summary our study suggests that the ASS enzyme is required to counterbalance the stress particularly during initial stage of infection when *L*. *donovani* parasites encounter oxidative stress. It is also required to maintain the virulence of *L*. *donovani* (AG83 strain). Further detailed investigations such as designing of novel inhibitor which specifically blocks LdASS activity without affecting the human counterpart or have minimal toxic effect on human ASS can establish it as a valid drug target for future chemotherapy for the treatment of visceral leishmaniasis.

The article "Genetic Manipulation of Leishmania donovani to Explore the Involvement of Argininosuccinate Synthase in Oxidative Stress Management" was retracted in 2023. Reasons: duplicated images; original data or images not available; unreliable data.

## Supporting Information

S1 Fig Western blot image of LdASS. The expression of LdASS protein was checked by Western blot analysis. The band corresponding to ~ 49 kDa (Lanes 1–6) shows the expression of LdASS. The lane denoted by “M” contains the protein molecular weight markers. The equal concentration of *L*. *donovani* cell lysate was loaded in lanes 1–6 and blot was developed by adding increasing concentration of rabbit serum containing polyclonal anti-LdASS (Lanes 1–6).
(TIF)

S2 Fig Western blot analysis of LdASS levels in *L*. *donovani* mutant cell lines. All the *L*. *donovani* cell lines recovered after a 4 week infection in BALB/c mice were examined by Western blot analysis to evaluate LdASS expression. No band was detected in LdASS -/-/+ cell lines whereas a faint and an overexpressed band (~ 49 kDa) was observed in LdASS-/+/+ and OE cell line compared to WT (LdASS+/+/+) cell lines.
(TIF)

S1 Table List of primers used in this study. (DOC)
